The article "Regulation of Quality of Life and Immune Function in Patients with Thyroid Cancer Treated by Deep Learning Technology" was retracted in 2023. Reasons: signs of a paper mill; suspected computer-generated content; unreliable results or conclusions; lack of ethics approval or compliance.

# Regulation of Quality of Life and Immune Function in Patients with Thyroid Cancer Treated by Deep Learning Technology

**DOI:** 10.1155/2022/3281039

**Published:** 2022-08-30

**Authors:** Xiandong Fu, Xinxin Yang, Yibo Wang, Nannan Chi, Jianan Yu, Yao Feng

**Affiliations:** ^1^Department of General Surgery, the First Affiliated Hospital of Jiamusi University, Jiamusi 154000, Heilongjiang, China; ^2^School of Clinical Medicine, Jiamusi University, Jiamusi 154000, Heilongjiang, China; ^3^Digestive Department, the First Affiliated Hospital of Jiamusi University, Jiamusi 154000, Heilongjiang, China; ^4^Department of Neurology, the First Affiliated Hospital of Jiamusi University, Jiamusi 154000, Heilongjiang, China; ^5^Traditional Chinese Medicine Department, the First Affiliated Hospital of Jiamusi University, Jiamusi 154000, Heilongjiang, China

## Abstract

**Background:**

In order to explore the regulation of quality of life and immune function in patients with thyroid cancer after radiotherapy, a method based on deep learning technology was proposed. A deep learning detection method for thyroid cancer is proposed.

**Methods:**

It mainly includes three main modules: data preprocessing, thyroid cancer regional detection module, and thyroid cancer benign and malignant classification module. The data set in the experiment comes from LIDC-IDRI and is processed by the data preprocessing module to generate a standard data format that can be processed by the framework. The treatment of thyroid cancer can help patients relapse malignant thyroid cancer and prevent recurrence in advance.

**Results:**

The results showed that most patients are diagnosed because of obvious swelling of local thyroid mass and conscious compression symptoms in the neck. At this time, they often miss the best treatment time, so as to reduce the surgical effect.

**Conclusions:**

The metastasis and invasion of cancer cells are fast, the cancerous lesions are easy to form adhesion with the surrounding tracheal tissue, and the cancer cells invade the surrounding soft tissue, which is also easy to cause the cancerous tissue not to be completely removed. *Clinical Trial Registration*. Therefore, deep learning technology is used to treat residual cancerous lesions to ensure the surgical effect.

## 1. Introduction

The incidence rate continues to increase. 56000 new thyroid cancers are projected every year in the United States. Thyroid cancer has become the fifth most common cancer in American women since 2010. Thyroid cancer is the second most common cancer among Italian women aged ≤45 years. In 2011, thyroid cancer ranked first in the ranking of cancer prevalence in Korea. In 2012, China's annual report of 32 cancer registry centers showed that thyroid cancer ranked fourth in city population, and the incidence rate increased by 14.5% [1] in 2003–2007 years. In 2010, the incidence rate of thyroid cancer in China was 4.1/10 million. The World Health Organization (who) estimates that there will be 48650 new cases of thyroid cancer in China in 2015. There are differences in survival status among countries. The latest survival data of thyroid cancer patients released by the United States, Europe, and China are as follows: SEER of the National Institutes of health in 2013 (surveillance, epidemiology, and end results program) released the survey data on the survival status of cancer patients, including 55834 patients diagnosed with thyroid cancer from 2003 to 2009 registered in 9 regions. All patients were followed up until 2010 [2]. The results showed that the 5-year relative survival rate of thyroid cancer patients (adjusted for race, gender, years of diagnosis, clinical stage, and age) was 98.2%, ranking the second among all cancers. According to previous literature reports, the five-year survival rate of thyroid cancer patients in the United States was only 64.0% in the 1940s, increased to 83.0% in the 1960s, and increased to 98.2% from 2003 to 2009. In the European cancer patient survival data released in 2014, a total of more than 10 million cancer patients in 107 cancer registries in 29 countries were included. All patients were diagnosed with cancer from 1999 to 2007. After follow-up to 2008, the age adjusted 5-year relative survival rate of thyroid cancer was 86.5% [3]. The relevant literature published in the UK in 2009 included patients diagnosed with cancer in 20 cancer registries from 1995 to 1999. After follow-up to 2003, the 5-year relative survival rate of thyroid cancer patients was 77.6%. In 2014, the data released by China Cancer Center showed that the 5-year relative survival rate of thyroid cancer was 67.5%, ranking second among all cancers. The statistics included 138852 patients first diagnosed with cancer from 2003 to 2005 recorded by 17 cancer registries, including 1736 cases of thyroid cancer. All patients were followed up to December 31, 2010 [4]. Data were collected through death records and dynamic follow-up (hospital medical records, medical insurance, and questionnaire), including 3 urban areas and 14 township areas, with the proportion of township areas close to 70%. According to the cancer statistics of China in 2015, there were nearly 90000 new cases of thyroid cancer, including 22000 males and 67900 females. There were 6800 deaths from thyroid cancer, including 2500 males and 4300 females. The incidence rate of thyroid cancer is first [5] in young women aged <30 years.

The article "Regulation of Quality of Life and Immune Function in Patients with Thyroid Cancer Treated by Deep Learning Technology" was retracted in 2023. Reasons: signs of a paper mill; suspected computer-generated content; unreliable results or conclusions; lack of ethics approval or compliance.

The concept of postoperative fatigue was first introduced in 1954 by Professor Merton. In 1978, two professors, Rose and King, systematically discussed that postoperative fatigue syndrome refers to a series of physical and mental problems, such as metabolic disorders, malnutrition, reduced immunity, and skeletal muscle contractility and decreased endurance. It is mainly manifested in the brain nervous system, cardiovascular system, skeletal muscle system fatigue, resulting in patients to fatigue, fatigue, insomnia, insomnia, tension, anxiety, and attention as the main manifestations of a group of symptoms, lasting up to 1–2 months. These are defined as a common group of signs after surgery and among the main complications of the postoperative recovery period. In recent years, the incidence of thyroid nodules is in a rapid growth trend, with the unexpected detection rate as high as 67%, and the incidence of thyroid malignant tumors in coastal cities increases with an average annual growth rate of 4%, which is one of the fastest growing malignant tumors. Surgery is widely recognized as the most important treatment method. Although most patients recover well after surgery, the trauma of surgery will lead many patients to show “postoperative fatigue syndrome,” and thyroid surgery intraoperative cervical overextension and shoulder high head low, combined with surgical injury, anesthetic drug stimulation, and other comprehensive factors induce patients in addition to the general postoperative fatigue syndrome. There will also be head, neck, shoulder, and back muscle pain, dizziness, headache, fatigue, shortness of breath, nausea and vomiting, and other symptoms. Therefore, some scholars refer to the thyroid surgery patients' postoperative fatigue, upset, anxiety, inattention, and other symptoms as “thyroid surgery postoperative fatigue syndrome.” Its incidence rate is very high, which is one of the common thorny problems in the postoperative rehabilitation process of thyroid patients. It will not only prolong the time of patients' postoperative discharge and return to normal life, but also reduce the short-term quality of life after surgery and even lead to patients not being able to return to normal work as soon as possible after surgery, which brings heavy economic burden to individuals and families.

In recent years, the treatment methods for thyroid tumors at home and abroad have been constantly updated, and the main treatments include surgery, endocrine drug therapy, iodine radiation therapy, and gene therapy. With the vigorous development of TCM and the enhancement of people's concept of TCM, more and more patients with thyroid tumors are more willing to try safe and effective TCM without obvious toxic and side effects. Therefore, it is of great significance to bring the characteristics of traditional Chinese medicine to the treatment of thyroid tumor patients as much as possible.

The article "Regulation of Quality of Life and Immune Function in Patients with Thyroid Cancer Treated by Deep Learning Technology" was retracted in 2023. Reasons: signs of a paper mill; suspected computer-generated content; unreliable results or conclusions; lack of ethics approval or compliance.

## 2. Literature Review

Taghiloo et al. [6] proposed a method combining local texture features and multiexample learning to extract local texture features from the region of interest, regard the region of interest as an example package composed of all local features, and finally use KNN algorithm to classify thyroid nodules, with an accuracy of 85.59% [6]. Tianyi et al. [7] introduced the binary regression model, took the benign and malignant of thyroid nodules as the dependent variable, took the ultrasonic performance as the independent variable, used logistic regression analysis to screen the ultrasonic indexes that can significantly distinguish the benign and malignant of thyroid nodules, and established the regression model, which has improved the accuracy. For the influence of spots in the image on the extracted features [7], Grigerová et al. [8] focused on studying and improving the thyroid tumor feature extraction algorithm. It overcomes the uncertainty of thyroid image classification caused by spots in thyroid ultrasound image. Finally, a new feature extraction method of thyroid ultrasound image combining texture, shape, and attenuation feature information is proposed, which has higher classification accuracy [8]. Based on the processing of large sample thyroid ultrasound images, Fu et al. [9] proposed a predictive association rule classification algorithm to deal with the mining of high-dimensional database. With the further development of association rules, other algorithms have emerged as auxiliary optimization methods. The improved dynamic integration algorithm based on *K*-means clustering 17 has good results. A selective weighted dynamic integration method is proposed. The parallel integration of multiple classifiers increases the stability of the classification model and proves a better classification algorithm than BP neural network [9]. Cheng et al. [10] combined the model of low-level features automatically extracted from images and high-level knowledge search from experts. The association rule technology based on Apriori algorithm improves the accuracy of good and evil classification after optimizing the objective function of graph theory [10, 11]. Jiang et al. [12] found that the local control rate of external radiotherapy group for papillary cancer was good, and the recurrence rate was reduced to 8%, compared with 25% in the control group. In Princess Margaret Hospital, Canada, 33 patients with differentiated thyroid cancer who received external radiotherapy had no recurrence for 5 years, and the local control rate was 62% [12]. The median overall survival time of 66 patients with differentiated thyroid cancer studied by Picardo et al. [13] was 42 months. Compared with patients with well and moderately differentiated thyroid cancer, the local control effect was significantly improved. The 3-year recurrence free survival rate in the nonadjuvant chemotherapy group was 73%, while that in the concurrent chemotherapy group was increased to 90% [13]. Pilla L. and Maccalli [14] reported that, in a group of 68 patients with tumor invading trachea undergoing tracheotomy, external radiotherapy significantly reduced local recurrence, and the recurrence rate decreased from 51% to 8% (*P* < 0.01) [14]. Drakes et al. [15] reported that the local control rate of a group of patients with differentiated thyroid cancer with positive surgical margin under microscope after external radiotherapy is 89.1%, and the local control rate of patients with naked eye residue or inoperable after external radiotherapy is 69.2% [15].

The article "Regulation of Quality of Life and Immune Function in Patients with Thyroid Cancer Treated by Deep Learning Technology" was retracted in 2023. Reasons: signs of a paper mill; suspected computer-generated content; unreliable results or conclusions; lack of ethics approval or compliance.

Based on the current research, as shown in Figure 1, a method based on deep learning technology is proposed. A deep learning detection method for thyroid cancer is proposed. It mainly includes three main modules: data preprocessing, thyroid cancer regional detection module, and thyroid cancer benign and malignant classification module.

## 3. Deep Learning Technology

In this paper, a deep learning detection method for thyroid cancer is proposed. The flow chart of the treatment method is shown in Figure 2, which mainly includes three main modules: data preprocessing, thyroid cancer area detection module, and thyroid cancer benign and malignant classification module. The data set in the experiment comes from LIDC-IDRI and is processed by the data preprocessing module to generate a standard data format that can be processed by the framework.

Before the neural network was proposed, when studying the brain, biological researchers found that the brain used a special processing mechanism for external information, namely, hierarchical processing [16, 17]. When the eye receives visual information, it transmits the information to the cerebral cortex. The information is transmitted and processed among multiple neurons and then transmitted to the next layer of neurons. It is hoped that the artificial neural network model can simulate this mechanism in the computer and process the information complex and effectively [18].

After surgery, the body was in a high metabolic state with negative nitrogen balance and significantly reduced protein. Therefore, postoperative nutritional support therapy can provide energy for the high metabolic status after surgery. A large number of experiments have proved that nutritional support therapy has a significant effect on accelerating postoperative recovery, especially when giving adequate nutrition to patients with severe postoperative undernutrition, which can significantly shorten the postoperative recovery time and accelerate the rapid recovery of patients to the preoperative physical fitness level. Branched-chain amino acids are one of the important raw materials for protein synthesis. And they are the source of energy when the body suffers from trauma and blood loss. After surgery, the decomposition of protein and muscle can be inhibited by supplementing branched chain amino acids, promote the synthesis of liver protein to correct the negative nitrogen balance of the body, and also reduce the ratio of free tryptophan to branched chain amino acids in plasma and improve postoperative fatigue. Oral administration of a high-dose concentration of carbohydrates before surgery can improve postoperative insulin resistance and reduce myosin breakdown, thus relieving postoperative fatigue.

The article "Regulation of Quality of Life and Immune Function in Patients with Thyroid Cancer Treated by Deep Learning Technology" was retracted in 2023. Reasons: signs of a paper mill; suspected computer-generated content; unreliable results or conclusions; lack of ethics approval or compliance.

After surgery, the body is in a state of stress, the hormone secretion in the body increases, the immune system activates, the body metabolism speed is significantly faster, and the protein content in the body is reduced, thus leading to the sense of fatigue in patients. In addition, preoperative fasting and other treatment result in the human body in a negative nitrogen balance state. Postoperative application of growth hormone can improve the conversion rate of nutrients, promote protein synthesis, and correct the negative nitrogen balance, which can effectively improve the postoperative fatigue symptoms of patients. Expert studies have found that the combination of growth hormone and nutritional support can reduce the duration of postoperative fatigue and reduce the degree of postoperative fatigue. Growth hormone also has the effect of promoting cell proliferation and inhibiting cell apoptosis, which may promote the growth of tumor cells, so the application in patients after tumor surgery is still controversial.

There are many examination methods that can be applied in the diagnosis of thyroid disease. For thyroid nodules with more than 1 cm in diameter, neck ultrasound is still the preferred examination method, which has the advantages of convenience, high accuracy, and high potency ratio. However, routine ultrasound is still difficult to distinguish between benign and malignant thyroid nodules, especially in the diagnosis of small carcinoma. Routine CT and MRI examination can further determine the thyroid nodule size and its relationship with adjacent tissues and organs, and the enhanced CT and MRI examination are helpful in the benign and malignant judgment of thyroid nodules. CT and MRI are feasible for further assessment of thyroid cancer that may invade the surrounding adjacent tissue or have multiple cervical lymph node metastases.

The article "Regulation of Quality of Life and Immune Function in Patients with Thyroid Cancer Treated by Deep Learning Technology" was retracted in 2023. Reasons: signs of a paper mill; suspected computer-generated content; unreliable results or conclusions; lack of ethics approval or compliance.

In the past few years, more and more scholars have begun to pay attention to the progress of the molecular biology of cancer, and the current widely recognized thyroid oncogene mutations are rat sarcoma strain toxic bacteria carcinogenic orthologs *B*1, RAS gene mutation, and BET/PTC rearrangement. In addition to tyrosine kinase receptor gene mutations and overexpression on the cell membrane, the abnormal activation of the downstream kinase pathway is also an important mechanism of thyroid cancer development and progression. Various related overexpression receptors including vascular endothelial growth factor (VEGF), epidermal growth factor (EGF), and platelet-derived growth factor (PDGF) make the thyroid potentially highly cancerous. Based on the molecular mechanisms, as well as the specific molecular targets of the tumorigenesis and growth process, the developed targeted drugs can bind to these targets and prevent or alleviate further tumor development. These include tyrosine kinase inhibitors (TKIs), cell growth factors and their receptor inhibitors, anti-VEGF drugs, EGF receptor inhibitors, DNA methylation inhibitors, cyclooxidase-2 receptors, and cell-cycle regulatory drugs. Several targeted therapeutics have been applied in the treatment of thyroid cancer, especially in recurrent and metastatic thyroid cancer. The drugs that have passed the phase of clinical experiments are mainly TKIs, and the representative drugs are serafini, vandetanib, pazopanib, and others. The clinical application data show that this drug has shown a good role in controlling tumor progression. Other types of targeted drugs, such as retinoic acid (RA), DNA methylation inhibitors, and histone deacetylase (HDAC) inhibitors, are currently in the research stage. Therefore, with the progress of the molecular biology of tumors, molecular targeted therapy will also play an important role in the treatment of thyroid cancer.

### 3.1. Forward Propagation

Neuron is the basic unit of neural network. The most basic structure of neuron is shown in Figure 3.

Neuron structure consists of four basic components: input, bias, activation function, and output. The input of the computer warp element in the figure can be expressed as an eigenvector *x*(*x*_1_, *x*_2_, *x*_3_), and the output value is

(1) $$\begin{array}{c} h_{W,b}\left(x\right)=f\left(W^{T}x\right)\text{,}\\ f\left(W^{T}x\right)=f\left(\overset{n}{\underset{i=1}{\sum }}W_{i}x_{i}+b\right)\text{,} \end{array}$$

where *W* is the weight matrix, *n* is the dimension of the input vector, and *f*(•) is the offset. *B* is the activation function of neurons. The input of neurons passes through the linear combination of *W* weight matrix, and the activation function introduces nonlinear factors into the model. If the network is shallow, when the activation function is a linear mapping relationship, and the linear weighted interaction between neurons is processed, the result is still a linear combination, which will reduce the expression ability of a certain model [19].

The article "Regulation of Quality of Life and Immune Function in Patients with Thyroid Cancer Treated by Deep Learning Technology" was retracted in 2023. Reasons: signs of a paper mill; suspected computer-generated content; unreliable results or conclusions; lack of ethics approval or compliance.

The neural network model takes neurons as the smallest unit, which are arranged and connected by neurons according to levels [20–22]. Each layer of neurons is output to the next layer of neurons after weighted combination of input data and activation function processing.  Figure 4 shows a simple feedforward neural network. The neural network consists of three parts: input layer *L*_1_, middle hidden layers *L*_2_, *L*_3_, and output layer *L*_4_. The input layer receives the incoming original feature vector, and all layers in the middle are hidden layers.

The input eigenvector *x*(*x*_1_, *x*_2_, *x*_3_) is calculated layer by layer through the neural network to produce the final output value, that is, the learning task of the network, output *h*_*w*,*b*_(*x*). Assuming that the output value of layer *L* processed by the activation function is *a*^(*l*)^, the weight matrix *W*^(*l*)^ is connected between layer *L* and the next layer *L* + 1, and the offset of layer *L* + 1 is *b*^(*l*)^, and the weighted sum result of layer *L* + 1 is vector *z*^(*l*+1)^, which has the following relationship:

(2) $$\begin{array}{c} z^{\left(l+1\right)}=W^{\left(l\right)}a^{\left(l\right)}+b^{\left(l\right)}\text{,}\\ a^{\left(l+1\right)}=f\left(z^{\left(l+1\right)}\right)\text{.} \end{array}$$

### 3.2. Backpropagation

The backpropagation algorithm has been proved to be good for training neural network model. The core step of the backpropagation algorithm is to calculate the data of the input layer and then inversely deduce the error of the output layer. In this way, the gradient of each parameter in the neural network is updated. The parameter update process is optimized by using the common gradient descent method [23].

Assuming that a data set {*x*^(*l*)^, *y*^(*l*)^, ..., *x*^(*m*)^, *y*^(*m*)^} with a sample number of *m* is given, the neural network is built to train and learn the sample data set, so that the neural network can well express the mapping relationship between input and output. Here, take the mean square error as an example to define the objective function:

(3) $$\begin{array}{c} J\left(A,c\right)=\left[\frac{1}{n}\overset{n}{\underset{t=1}{\sum }}J\left(A,b;x^{\left(t\right)},y^{\left(t\right)}\right)\right]+\frac{\gamma }{2}{\overset{m_{t}-1}{\underset{p=1}{\sum }}\overset{s_{p}}{\underset{t=1}{\sum }}\overset{s_{p}+1}{\underset{f=1}{\sum }}\left(A_{ft}^{\left(p\right)}\right)}^{2}\text{,}\\ J\left(A,c\right)=\left[\frac{1}{n}\overset{n}{\underset{t=1}{\sum }}\left(\frac{1}{2}{\left\|h_{A,c}\left(x^{\left(t\right)}\right)-y^{\left(t\right)}\right\|}^{2}\right)\right]+\frac{\lambda }{2}{\overset{m_{t}-1}{\underset{p=1}{\sum }}\overset{s_{p}}{\underset{t=1}{\sum }}\overset{s_{p}+1}{\underset{f=1}{\sum }}\left(A_{ft}^{\left(p\right)}\right)}^{2}. \end{array}$$

The first part is the mean square deviation term, and the second part is the regular term. By increasing the regular term, the overfitting of the model can be effectively reduced. The parameter optimization method in neural network usually adopts batch gradient descent, random gradient descent, Adam, and other methods. Here, taking batch gradient descent as an example, each parameter in neural network is updated iteratively, where *α* is the learning rate [24], which is used to adjust the “step size” of model learning:

(4) $$\begin{array}{c} A_{ft}^{p}=A_{ft}^{p}-\alpha \frac{\partial }{\partial A_{t}^{\left(p\right)}}J\left(A,c\right)\text{,}\\ c_{ft}^{\left(p\right)}=c_{ft}^{\left(p\right)}-\alpha \frac{\partial }{\partial A_{t}^{\left(p\right)}}J\left(A,c\right)\text{.} \end{array}$$

The parameter updating method in neural network first needs to calculate the partial derivative of the objective function formula to each parameter and then use the backpropagation algorithm to update the parameters. The specific steps are as follows:

(1) Firstly, the forward propagation algorithm is used to calculate the hidden layers *L*_2_, *L*_3_ in the neural network. After receiving the input, the result in the output layer *L*_*nl*_ is obtained through the action of the activation function.
(2) Then, calculate the residual *δ*_*i*_^(*nl*)^ between the output layer result and the real value:
  (5) $$\begin{array}{c} \delta_{i}^{\left(nl\right)}=\frac{\partial }{\partial z_{i}^{\left(nl\right)}}\frac{1}{2}{\left\|y-h_{W,b}\left(x\right)\right\|}^{2}\text{,}\\ \delta_{i}^{\left(nl\right)}=-\left(y_{i}-a_{i}^{\left(nl\right)}\right)\cdot f^{\prime }\left(z_{i}^{\left(nl\right)}\right)\text{.} \end{array}$$
(3) Calculate the reverse derivation process; that is, calculate the residual value of the hidden layer of the neural network, and calculate the derivation from back to front step by step:
  (6) $$\begin{array}{c} \delta_{i}^{\left(l\right)}=\left(\overset{s_{t+1}}{\underset{j=1}{\sum }}W_{ji}^{\left(l\right)}\delta_{j}^{\left(l+1\right)}\right)f^{\prime }\left(z_{i}^{\left(l\right)}\right)\text{.} \end{array}$$
(4) Finally, the final partial derivative is obtained by using the residual value calculated in the previous steps:
  (7) $$\begin{array}{c} \frac{\partial }{\partial W_{ij}^{\left(l\right)}}J\left(W,b;x,y\right)=a_{j}^{\left(l\right)}\delta_{i}^{\left(l+1\right)}\text{,}\\ \frac{\partial }{\partial W_{i}^{\left(l\right)}}J\left(W,b;x,y\right)=\delta_{i}^{\left(l+1\right)}\text{.} \end{array}$$

The article "Regulation of Quality of Life and Immune Function in Patients with Thyroid Cancer Treated by Deep Learning Technology" was retracted in 2023. Reasons: signs of a paper mill; suspected computer-generated content; unreliable results or conclusions; lack of ethics approval or compliance.

### 3.3. Preprocessing Data

The data preprocessing process is shown in Figure 5 mainly including connected area analysis, data cutting, and data enhancement. The specific flow is as follows.

#### 3.3.1. Connected Region Analysis

There are many fragmentary outliers in the image recognized by the thyroid cancer detection module. These outliers may belong to the same thyroid cancer region, so the necessary connectivity region analysis needs to be carried out, and all detected thyroid cancer candidate regions need to calculate the nodule center of the candidate thyroid cancer. The adjacency relationship is generally divided into 4-adjacency relationship and 8-adjacency relationship. This experiment adopts the 8-adjacency relationship; that is, one of the 8 adjacent pixels around each pixel is adjacent to another connected region, that is, the pixel is considered to belong to the connected region [25–27]. After expansion operation and 8-adjacent connected region labeling, the number of candidate thyroid cancers can be reduced, the adjacent small thyroid cancers can be combined, the experimental cost can be saved, and the repeated recognition and classification of regions with high repetition rate can be avoided.

#### 3.3.2. Data Cutting

The classification of benign and malignant thyroid cancer is essentially an image classification problem. The test is based on the detection of thyroid cancer. The candidate thyroid cancer area after thyroid cancer detection is 64 × sixty-four × 64. The diameter of thyroid cancer is defined as 3–30 mm. Generally, the diameter of thyroid cancer is about 10 mm. Therefore, in order to enable the model to more accurately extract the features of the thyroid cancer image region in the classification process and reduce the unnecessary amount of calculation, the experimental process takes the candidate thyroid cancer as the center and cuts 32 × thirty-two × 32 3D image data [28, 29]. Assuming that the central coordinates of thyroid cancer are (*x*, *y*, z), the volume of 3D image data cut *V*(*x* − *d* : *x*+*d*, *y* − *d* : *y*+*d*, *z* − *d* : *z*+*d*), where *d* represents half of the side length of 3D cube data, i.e., *d* = 16. In particular, when thyroid cancer is at the edge, it is necessary to detect the boundary of the cube to prevent it from exceeding the visible range of the image.

The article "Regulation of Quality of Life and Immune Function in Patients with Thyroid Cancer Treated by Deep Learning Technology" was retracted in 2023. Reasons: signs of a paper mill; suspected computer-generated content; unreliable results or conclusions; lack of ethics approval or compliance.

### 3.4. Experimental Methods

The control group received routine nursing, mainly including the following:

1. Cognitive behavior education: educate patients and their families on the etiology, pathogenesis, and treatment of thyroid cancer, so that patients have a correct understanding of the disease and reduce their wrong understanding of the disease;
2. Psychological nursing: nurses should understand the psychological state of patients, observe their daily living habits, actively communicate with patients, and listen patiently, carry out targeted psychological counseling for patients, encourage patients to communicate more with roommates and family members, improve patients' psychological comfort, targeted emotional adjustment, and psychological intervention, and eliminate patients' bad emotions;
3. Dietary guidance: ask to choose light and digestible foods with high protein, high calories, and high vitamins. Sometimes, the diet is frugal, and carry out activities with certain tolerance after meals [30, 31];
4. Chemotherapy guidance: educate patients on chemotherapy related knowledge, emphasize that standardized chemotherapy can prolong the survival cycle, and inform them of the treatment of related toxic and side effects.

### 3.5. Observation Indicators

Changes of immune function: all patients took blood before and after nursing to check the changes of immune indexes such as CD3+, CD4+, and CD8+.

1. Anonymous questionnaire was used to evaluate the satisfaction rate of patients, and Likert questionnaire and scoring were used for statistics;
2. The compliance was evaluated by the medical staff, and then the evaluation results were integrated into three grades: better, average, and poor. The incidence of compliance = (better +average)/total number of cases ×  100%. After radiotherapy, the two groups were followed up in detail. The Chinese version of the core scale for cancer patients (eortcqlc-c30) was used to investigate the quality of life [32, 33]. There are 30 items in this scale.

## 4. Results and Analysis

### 4.1. Comparison of Immune Function Changes between the Two Groups

After chemotherapy, CD3 + and CD4 + in the two groups increased and CD8 + decreased, while the immune indexes of the treatment group changed significantly compared with the control group (*P* < 0.05) (see Figures 6–9).

The article "Regulation of Quality of Life and Immune Function in Patients with Thyroid Cancer Treated by Deep Learning Technology" was retracted in 2023. Reasons: signs of a paper mill; suspected computer-generated content; unreliable results or conclusions; lack of ethics approval or compliance.

### 4.2. Comparison of Satisfaction Rate and Compliance between the Two Groups

After nursing, the satisfaction rate of the treatment group was 100.0%, which was higher than 50% of the control group, and the difference was statistically significant (*P* < 0.05) (see Figures 10 and 11).

### 4.3. Quality of Life (Functional Area) Score

The quality of life (functional area) score of the treatment group was higher than that of the control group, and the difference was statistically significant (*P* < 0.05) (see Figures 12 and 13).

### 4.4. Comparison of Quality of Life (Overall Health + Symptom Area) Scores between the Two Groups

The overall health score of patients in the treatment group was higher than that in the control group, while the symptom score was lower than that in the control group, suggesting that the improvement of quality of life of patients in the treatment group was better than that in the control group (*P* < 0.05) (see Figures 14 and 15).

Therefore, there is postoperative cancer cell proliferation or recurrence, which reduces the clinical curative effect and endangers life. Patients with thyroid cancer have no specific clinical manifestations in the early stage. At this time, they often miss the best treatment time, so as to reduce the surgical effect. The metastasis and invasion of cancer cells are fast, the cancerous lesions are easy to form adhesion with the surrounding tracheal tissue, and the cancer cells invade the surrounding soft tissue, which is also easy to cause the cancerous tissue not to be completely removed. Therefore, deep learning technology is used to treat residual cancerous lesions to ensure the surgical effect [34]. At the same time of effective treatment, radiotherapy lacks selective killing effect, so inhibiting tumor cells can also damage normal immune active cells such as granulocytes, lymphocytes, and macrophages. At this time, it can also damage proliferating epithelial cells such as gastrointestinal epithelial cells and germ cells. Therefore, during radiotherapy, patients often suffer from nausea, vomiting, anorexia, and other discomfort, resulting in malnutrition and low body resistance in most patients during postoperative recovery, and finally patient compliance is reduced. Therefore, effective nursing intervention during radiotherapy and after discharge is of great significance to the postoperative recovery of patients. Deep learning technology nursing intervention is an open and extended health education method completed by information means, which aims to improve the quality of life of discharged patients and improve treatment compliance. By strengthening the contact between nurses and patients and their families, we can escort patients' health care. After continuation and development, it has been widely used in cancer patients. Through regular telephone follow-up and home visits, strengthen patients' cognition of the disease, reduce misunderstanding of cancer, and eliminate resistance and worry about radiotherapy [35]. During radiotherapy, patients' bad emotions such as anxiety and depression can be relieved, and timely encouragement and education can establish their recovery confidence. By strengthening the contact and interaction between patients and their families, the emotional support of patients can be enhanced.

The article "Regulation of Quality of Life and Immune Function in Patients with Thyroid Cancer Treated by Deep Learning Technology" was retracted in 2023. Reasons: signs of a paper mill; suspected computer-generated content; unreliable results or conclusions; lack of ethics approval or compliance.

## 5. Conclusion

To sum up, the nursing effect of deep learning technology on patients with thyroid cancer undergoing radiotherapy is satisfactory, which can effectively improve the quality of life of patients during and after radiotherapy and improve the immune function of distant body. It is worthy of clinical application.

## Figures and Tables

**Figure 1:** Deep Learning Technology in the treatment of thyroid cancer.

**Figure 2:** Flowchart of thyroid cancer detection method based on deep learning.

**Figure 3:** Basic structure of neurons.

**Figure 4:** Feedforward neural network.

**Figure 5:** Flow chart.

**Figure 6:** Comparison of immune function before radiotherapy in the treatment group.

**Figure 7:** Comparison of immune function after chemotherapy in the treatment group.

**Figure 8:** Comparison of immune function in the control group before radiotherapy.

**Figure 9:** Comparison of immune function in the control group after chemotherapy.

**Figure 10:** Comparison of compliance between the two groups.

**Figure 11:** Comparison of patient satisfaction between the two groups.

**Figure 12:** Evaluation of quality of life in the treatment group.

**Figure 13:** Quality of life evaluation of control group.

**Figure 14:** Quality of life of patients in the treatment group (comparison of scores in overall health + symptom area).

**Figure 15:** Quality of life of patients in the control group (comparison of scores in overall health + symptom area).

## Data Availability

The data that support the findings of this study are available from the corresponding author upon reasonable request.
